# The Classification of Music and Art Genres under the Visual Threshold of Deep Learning

**DOI:** 10.1155/2022/4439738

**Published:** 2022-05-18

**Authors:** Zhiqiang Zheng

**Affiliations:** School of Music, Henan Vocational Institute of Arts, Zhengzhou, Henan, China

## Abstract

Wireless networks are commonly employed for ambient assisted living applications, and artificial intelligence-enabled event detection and classification processes have become familiar. However, music is a kind of time-series data, and it is challenging to design an effective music genre classification (MGC) system due to a large quantity of music data. Robust MGC techniques necessitate a massive amount of data, which is time-consuming, laborious, and requires expert knowledge. Few studies have focused on the design of music representations extracted directly from input waveforms. In recent times, deep learning (DL) models have been widely used due to their characteristics of automatic extracting advanced features and contextual representation from actual music or processed data. This paper aims to develop a novel deep learning-enabled music genre classification (DLE-MGC) technique. The proposed DLE-MGC technique effectively classifies the music genres into multiple classes by using three subprocesses, namely preprocessing, classification, and hyperparameter optimization. At the initial stage, the Pitch to Vector (Pitch2vec) approach is applied as a preprocessing step where the pitches in the input musical instrument digital interface (MIDI) files are transformed into the vector sequences. Besides, the DLE-MGC technique involves the design of a cat swarm optimization (CSO) with bidirectional long-term memory (BiLSTM) model for the classification process. The DBTMPE technique has gained a moderately increased accuracy of 94.27%, and the DLE-MGC technique has accomplished a better accuracy of 95.87%. The performance validation of the DLE-MGC technique was carried out using the Lakh MIDI music dataset, and the comparative results verified the promising performance of the DLE-MGC technique over current methods.

## 1. Introduction

Music in vast collections is becoming increasingly difficult to find, browse, and suggest. It is mandatory to maintain all of the tags linked with a piece of music to make it easier for others to find the requirement. Annotations can be added either manually or automatically [1]. On the other hand, the amount of necessary human labor is prohibitively expensive for manual annotation operations. It is possible to categorize songs, albums, and artists based on their shared musical traits by applying genre designations to their work. Music genres have long been used to sort music into various subgenres [2]. A hot topic of discussion has arisen because of this: automated music genre categorization. Numerous academics categorize music into broad genres (such as Pop or Rock) utilizing handmade audio elements and assigning a single label to each track [3]. Several issues arise with this proposal. First, it should be noted that not all musical subgenres are mutually incompatible. For example, a song that incorporates parts of Deep House and Reggae may be labeled as Pop (eSongs that are Pop but also have aspects of Deep House and Reggae rhythm might be considered hybrids) [4]. Second, the variability of the data may not be well represented by the characteristics that have been developed. Representational learning strategies have consistently outperformed all others when it comes to learning. It is also possible to identify genres using a broad range of data from audio, images, and text [5]. There is a range of ways to deal with various types of modalities. This music information retrieval (MIR) problem, which involves both single-label and multilabel categorization, does not yet have a deep learning multimodal technique, as far as we are aware.

We offer a system that can accurately predict music genre labels [6]. We employ a two-pronged approach: A neural network is used to teach the categorization job for each modality. In a multimodal technique, intermediate representations are retrieved and concatenated from each network. Experiments on single-label and multilabel genre categorization are used to test the effects of the newly discovered data representations and their combination [7]. It is possible to train convolutional neural networks on spectrogram data, encoding audio signals as time-frequency representations (CNNs). Album cover photographs are used to train an advanced convolutional neural network (CNN) pretrained using parameters learned in a generic image classification task and then fine-tuned to classify music genre labels [8]. Representations of texts from music-related publications are learned by feeding forward networks across a Vector Space Model (VSM) that has been augmented with semantic information using Entity Linking (EL). This information is the first time audio and visuals have been utilized to test single-label classification [9]. A multimodal feature space may be learned by matching a given dataset's visual and aural data representations. Using an auditory-visual method to categorize items is more successful than alone using either an audio or visual strategy [10]. Despite the absence of visual data, multimodal feature space enhances auditory representations. Using human annotator results as a benchmark, we analyze how well our trained algorithms categorize images. These results show how well the combined audio and visual representations work [11]. This study looks at different parts of the input photographs to see how the deep visual model judges each genre. These results were confirmed in an experiment that combined audio, text, and graphics to create a multilabel classification system [12]. Better scores are achieved when many modes of data acquisition are combined. The results demonstrate that deep neural networks outperform a traditional audio-based technique that relies on handcrafted characteristics. Deep learning architectures for audio categorization are also compared in a comprehensive manner [13]. An increased dimensionality reduction approach is used for labels in this comparison. The experiment's multilabel categorization is then thoroughly analyzed in terms of its quality [14]. An audio feature such as MFCCs is generally used to input a machine learning classifier in classical techniques, such as neural networks and deep neural networks [15]. Spectrograms, which are visual representations of an audio stream, have been used in recent deep learning algorithms [16]. A similar approach to picture categorization is used to feed these visual representations of audio into Convolutional Neural Networks (CNNs).

For this goal, researchers also looked at text-based approaches. In an early attempt to categorize music reviews, for example, work on multi-class genre categorization and star rating prediction is mentioned. Using an innovative method for predicting how people would use music, known as agglomerative clustering, they discovered that bigram characteristics were more informative than unigram features in their research [17]. Thus, POS tags and pattern mining techniques are employed to extract descriptive patterns for discriminating between positive and negative reviews. The meaning of a song can be deduced from its lyrics and other textual data, making it possible to predict its theme (e.g., love, war, or drugs). Album reviews use an SVM classifier to enrich and categorize them into 13 different genres [18]. Music genre classification with visuals is a relatively new field of study. Audio and song lyrics have frequently been used in studies of multimodal approaches [19]. Aside from text, music and video have also been considered. McKay and Fujinaga use cultural, symbolic, and auditory characteristics to categorize music. Other fields have done a lot of work on multilabel classification. In the framework of MIR, machine learning and deep learning have been used to study multilabel tag classification from audio (autotagging). It is challenging to classify music genres using multilabels since none of the algorithms employ representation learning or multimodal data [20].

More than 100,000 songs have been made available online since music streaming services were introduced. Genre-based playlists are the most crucial feature of these services. It is impossible to define exactly what goes into making a genre of music, although there are some commonalities among the music that falls under that category. Musical compositions can be categorized based on these characteristics. Even if music publishers create these labels, they do not serve any purpose in classifying music [21]. As the Internet and multimedia technologies have grown more widely available and popular, musical pieces have increased considerably in recent years. Professionals have been increasingly ineffectual in their role as the primary source of information for assessing and categorizing. Using software to classify music genres can significantly reduce the workload of human experts while also increasing the accuracy of the results [22].

K-Nearest Neighbor (KNN) and Support Vector Machine (SVM) are two of the most often used machine learning algorithms, Mixture Models, etc., that can solve the challenge of categorizing music genres. The performance of the conventional machine learning algorithm does typically not improve if the amount of data input exceeds a certain threshold. Deep learning algorithms, in particular, have gotten a lot of attention in the last several years. The complexity of feature engineering in traditional machine learning is more significant than that in deep learning. It is possible to reduce the amount of data needed to train machine learning algorithms by using feature engineering, which involves constructing feature extractors based on domain knowledge [23]. For example, if you label your data, you do not create a new feature extractor for each task. The accuracy of feature extraction is more important than the input volume for most machine learning algorithms in computer vision and natural language processing. Many different industries are now able to benefit from deep learning. As a result of the deep learning method, significant progress has been made in computer vision and natural language processing. As a result, MIR still has a long way to go compared to the two categories before it. As a result, researchers in MIR are increasingly turning to deep learning approaches to tackle their difficulties. A significant reduction in professional burden and an increase in industry-related application efficiency are possible outcomes of this implementation method. A solid basis and new ideas are presented to help solve more complex MIR issues [24].

Approaches such as the ones listed above have regularly surpassed the competition for classifying music into various genres. These strategies have yet to address how middle-level learning features influence the classification results of a complete model. Here, middle-level learning, which refers to the characteristics of other layers between an input and a classifier used for learning, is especially significant. The following has been simplified for clarity's sake. It is possible to use final learning features derived from a single input model or a multifeature model to classify data. It is assumed that other forms of learning are also involved in this interaction since the bottom learning feature is more beneficial than the top learning feature when taken into account. Middle-level learning feature interaction (MLFI) has been proposed to investigate this issue. The study focused on the classification of music and art genres under the visual threshold of deep learning. This paper is organized into four sections.  Section 1 presents the introduction and objectives of the study.  Section 2 highlights the methods used in the study.  Section 3 presents the results and analysis, and Section 4 focuses on the conclusion and future work.

The contributions of the study are as follows.

- This paper focuses on developing a novel deep learning-enabled music genre classification (DLE-MGC) technique.
- The proposed DLE-MGC technique effectively classifies the music genres into multiple classes by using three subprocesses, namely preprocessing, classification, and hyperparameter optimization.
- At the initial stage, the Pitch to Vector (Pitch2vec) approach is applied as a preprocessing step where the pitches in the input musical instrument digital interface (MIDI) files are transformed into the vector sequences.

## 2. Materials and Methods

Music genres are classifications of music based on the style of the music played by the players depending on the circumstances or storyline. In this work, experimental analysis is carried out on the Lakh MIDI music dataset, a highly reliable dataset commonly used for music genre classification. It includes a set of 176,581 MIDI files. This dataset was matched and aligned to entries in the Million Song Dataset. Amongst the Lakh MIDI dataset, 11,946 MIDI files have genre labels that comprise 13 class labels, namely, Pop/Rock, Electronic, Country R and B, Jazz, Latin, International, etc. In this work, a new DLE-MGC technique has been developed to detect and classify music genres. The proposed DLE-MGC technique incorporates three subprocesses, namely Pitch2vec-based preprocessing, BiLSTM based classification, and CSO-based hyperparameter optimization. The design of the CSO algorithm helps to appropriately tune the hyperparameters involved in the BiLSTM model.

### 2.1. Pitch2vec-Based Preprocessing

Primarily, the Pitch2vec approach is employed as a preprocessing step where the input MIDI files are transformed into vector sequences before passing into the BiLSTM model. At the time of Pitch2vec preprocessing, many asynchronous tracks exist in a MIDI file. When playing MIDI files, these tracks play varying roles, comprising one melody track, many chord tracks, and a drum track. For the standardization of the number of MIDI tracks, many chord tracks undergo syncretization into a single MIDI track. Pitch2vec Converter utilizes the pitch data and its respective index to derive pitch vectors. After the traversal of every MIDI file, the possible pitch combinations are obtained and filtered based on the frequency of the pitch combinations.

### 2.2. BiLSTM-Based Classification

During the classification process, the BiLSTM model receives the vector sequences and allots proper class labels to them. Long short term memory (LSTM) network is a kind of recurrent neural network (RNN) originally developed to resolve the gradient vanishing problems of RNN while handling longer sequences. An LSTM network structure comprises a standard feedforward network and layer of LSTM units. Generally, an LSTM unit functions as follows: consider *x*_*t*_ representing the existing input at time *t*, the output of the input gate,

(1) $$\begin{array}{c} i_{t}=\sigma \left(W_{i}^{x}x_{t}+W_{i}^{h}h_{t-1}+b_{i}\right), \end{array}$$

where *W*_*i*_^*x*^ and *W*_*i*_^*h*^ represent weight matrices, *h*_*t*−1_ denotes the preceding hidden layer of the unit, and *b*_*i*_ shows the bias vector. The function *σ*(*x*) ∈ (0,1) is a sigmoid function utilized for gating. Likewise, the output of forget gate *f*_*t*_ is calculated by

(2) $$\begin{array}{c} f_{t}=\sigma \left(W_{f}^{x}x_{t}+W_{f}^{h}h_{t-1}+b_{f}\right). \end{array}$$

Finally, the output of the output gate 0_*t*_ and cell state *c*_*t*_ are

(3) $$\begin{array}{c} c_{t}=i_{t}⊙\text{tanh}\left(W_{c}^{x}x_{t}+W_{c}^{h}h_{t-1}+b_{c}\right)+c_{t-1},\\ {\text{o}}_{t}=\sigma \left(W_{0}^{x}x_{t}+W_{0}^{h}h_{t-1}+b_{0}\right),\\ h_{t}={\text{o}}_{t}⊙\text{tanh}\left(c_{t}\right). \end{array}$$

in which, ⊙ represent the Hadamard product. The BiLSTM contains two similar LSTM layers: forward direction and backward direction, as shown in Figure 1. Since the input is processed two times, BiLSTM extracts further data from the input, therefore, enhancing contextual data for making effective predictions when compared to LSTM. Thus, BiLSTM presents fast accuracy and convergence when compared to LSTM. The BiLSTM framework consists of keeping past and future context at any time of the sequence. The output of LSTM is integrated as follows:

(4) $$\begin{array}{c} y_{t}=W_{\overset{⟶}{h}y}\overset{⟶}{h_{t}}+W_{\overset{\leftarrow }{h}y}\overset{\leftarrow }{h_{t}}+b_{y\prime }, \end{array}$$

where $\overset{⟶}{h_{t}}\text{ and }\overset{\leftarrow }{h_{t}}$ represent the output of forward and backward LSTM.

### 2.3. CSO-Based Hyperparameter Optimization

At the final stage, the CSO algorithm has been employed to tune the hyperparameter values of the BiLSTM model and thereby enhance the overall classification outcomes. The main advantage of the hyperparameter optimization in the machine learning algorithm is to provide the best performance by finding the hyperparameters which are measured based on the validation set. The CSO is a population‐based, comparatively stochastic, metaheuristic evolutionary approach. CSO imitates two natural behaviors of cats: tracing the targets and looking around their environments for the next move. They often stay alert even while at rest. They have excellent hunting skills and stronger inquisitiveness toward moving objects. One significant feature of cats is that they save their energy for future chasing and spend most of their time in inertia. In normal times, their movement is also slower. Once they sense prey, it chases very fast, spending massive energy. The CSO relates to; pursuing with high energy and speed as tracing mode and resting with slower movement as seeking mode. The increasing speed in the seeking process is arithmetically mapped as a significant change in the cat's position.

#### 2.3.1. Seeking Mode

There are five operators in the seeking mode: Seeking Range of Selected Dimension (SRD), Counts of Dimension to Change (CDC), Seeking Memory Pool (SMP), Mixture Ratio (MR), and Self-Position Consideration (SPC).

SRD is utilized to state the mutation part for the selected dimension. When the candidate a dimension is carefully chosen for mutation, the variance among the new and old values may not be out of range. CDC corresponds to the number of dimensions to be changed in the seeking method. SMP defines the number of copies of a cat produced or pool size of seeking memory when the values of SMP are set as 10. Then it is capable of storing ten solutions set as candidates. MR is a smaller value than the fraction of the population to guarantee that the cat spends its time seeking. SPC is a Boolean value, and when it is true, one position within the memory would store the existing solution set and remain unchanged. The steps implemented in the seeking process are given below.

  Step 1: number of cats that is *N* is formed by initializing the velocities, flag, and position of cat.
  Step 2: select some cats and based on the MR implement them to seeking and tracing modes.
  Step 3: estimate the fitness value according to its position.
  Step 4: when the end criterion is satisfied, the last solution would be the optimal position of the cat in the solution space. Or else, return to Step 2.

#### 2.3.2. Tracing Mode

It is exactly the same as the local searching model of the swarm in the PSO approach. In this process, the cat traces the target with higher energy by changing the position with its own velocity. The velocity and position of the *ith* cat in *D* dimension solution space are as follows:

(5) $$\begin{array}{c} X_{i}=\left[X_{i1},X_{i2},X_{i3},\ldots ,X_{iD}\right],\\ V_{i}=\left[y_{i1},y_{i2},y_{i3},V_{iD}\right]. \end{array}$$

The global optimal position of CSO is given by

(6) $$\begin{array}{c} g\text{best}=\left[g{\text{best}}_{1},g{\text{best}}_{2},\ldots ,g{\text{best}}_{D}\right]. \end{array}$$

Upgrade the position and velocity of the existing cat by utilizing equations (7) and (8):

(7) $$\begin{array}{c} V_{iD}=w*V_{iD}+c_{1}*r_{1}*\left(g{\text{best}}_{D}-X_{iD}\right), \end{array}$$

(8) $$\begin{array}{c} X_{iD}=X_{iD}+V_{iD}, \end{array}$$

where *w* represents the inertia weight, *c*_1_ denotes the acceleration constant, and *r*_1_ indicates an arbitrary value uniformly distributed within (0,1). A small inertia weight facilitates local searching while a large inertia weight helps global searching. In the work, *w* is fixed as 0.4. A cat swarm characterizes a set of indices. By utilizing this index, a reduced feature subset is acquired from the novel data set. It might take place during the selection more than one number of indices that may not fall (rare cases) in the range of column presented on the data set. For getting optimum candidate features with good classification performance, adapted CSO is employed for each dataset.

## 3. Results and Discussion

This section investigates the classification result analysis of the DLE-MGC technique on the benchmark dataset. The classifier results of the DLE-MGC technique are examined under two different epochs, namely, 1000 and 2000.  Table 1 and Figure 2 demonstrate the overall classification result analysis of the DLE-MGC technique under distinct classes and 1000 epochs. The table values indicated that the DLE-MGC technique has reached effective classification results under all classes. For instance, under Pop/Rock class, the DLE-MGC technique has obtained a precision of 94.87%, recall of 93.86%, F-score of 94.70%, and accuracy of 95.87%.

Concurrently, under the Electronic class, the DLE-MGC methodology has reached a precision of 93.17%, recall of 95.60%, F-score of 96.27%, and accuracy of 93.56%. Simultaneously, under the Rap class, the DLE-MGC algorithm has gained a precision of 96.45%, recall of 97.12%, F-score of 96.01%, and accuracy of 97.06%. Meanwhile, under the Blues class, the DLE-MGC method has reached a precision of 94.94%, recall of 95.46%, F-score of 96.41%, and accuracy of 94.27%.

Table 2 and Figure 3 showcase the overall classification outcome analysis of the DLE-MGC approach under various classes and 2000 epochs. The table values indicated that the DLE-MGC system has reached effectual classification outcomes under all classes. For instance, under the Pop/Rock class, the DLE-MGC method has reached a precision of 95.98%, recall of 95.58%, F-score of 97%, and accuracy of 95.98%. Concurrently, under the Electronic class, the DLE-MGC approach has attained a precision of 94.42%, recall of 96.51%, F-score of 97.32%, and accuracy of 96.14%. Simultaneously, under the Rap class, the DLE-MGC approach has reached a precision of 96.93%, recall of 95.51%, F-score of 97.43%, and accuracy of 95.72%. Meanwhile, under the Blues class, the DLE-MGC methodology has achieved a precision of 94.27%, recall of 95.29%, F-score of 95.91%, and accuracy of 94.64%.

The accuracy outcome analysis of the DLE-MGC approach on the test data is demonstrated in Figure 4. The outcomes exhibited that the DLE-MGC technique has accomplished enhanced validation accuracy related to training accuracy. It can also be observable that the accuracy values obtained saturated with the epoch count of 2000.

The loss outcome analysis of the DLE-MGC system on the test data is illustrated in Figure 5. The figure portrayed that the DLE-MGC technique has denoted the lower validation loss on the training loss. It can be additionally observed that the loss values attain saturated with the epoch count of 2000.

An average classification result analysis of the DLE-MGC technique under varying epochs is in Table 3. The table values showed that the DLE-MGC technique had obtained maximum classification performance. For instance, with 1000 epochs, the DLE-MGC technique has offered a precision of 94.97%, recall of 95.97%, F-score of 96.53%, and accuracy of 95.42%. Likewise, with 2000 epochs, the DLE-MGC method has obtainable precision of 95.84%, recall of 95.93%, F-score of 96.71%, and accuracy of 95.87%.

In order to highlight the enhanced music genre classification results of the proposed DLE-MGC technique, a comparative accuracy analysis is made in Table 4 and Figure 6. The results exhibited that the Two-LSTM and P2-PQA techniques have obtained worse outcomes with the minimal accuracy of 64.88% and 64.10% respectively.

At the same time, the DBTMPE technique has gained a moderately increased accuracy of 94.27%. However, the DLE-MGC technique has accomplished a better accuracy of 95.87%. From the abovementioned tables and figures, it is ensured that the DLE-MGC technique has the ability to achieve maximum music genre classification results compared to other techniques.

## 4. Conclusions

Artificial intelligence-enabled event detection and classification techniques are becoming commonplace in ambient assisted living applications. A compelling music genre classification (MGC) system cannot be designed because of the vast amount of data in the music industry. Using robust MGC approaches requires more data that will take a long time to collect and analyze. The design of music representations taken directly from input waveforms has received little attention due to their ability to automatically extract advanced features and contextual representations from actual music or processed data. Deep learning-enabled music genre classification (DLE-MGC) is developed due to this motivation. Three subprocesses, including preprocessing, classification, and hyperparameter optimization, are used in the proposed DLE-MGC technique to classify music genres into numerous classes effectively. Pitch to Vector (Pitch2vec) is used as a preprocessing step to convert the input musical instrument digital interface (MIDI) files' pitches into vector sequences. The DLE-MGC method utilizes a cat swarm optimization (CSO) model equipped with bidirectional long-term memory (BiLSTM) for the classification process. According to the experimental results, the proposed model has provided an accuracy of 95.87%. For future direction, it is highly recommended to implement the hybrid model for analyzing the genres in music.

## Figures and Tables

**Figure 1:** Structure of the BiLSTM model.

**Figure 2:** Result analysis of DLE-MGC technique under different music genre classes and 1000 epochs.

**Figure 3:** Result analysis of the DLE-MGC technique under different music genre classes and 2000 epochs.

**Figure 4:** Accuracy graph analysis of DLE-MGC technique under 2000 epochs.

**Figure 5:** Loss graph analysis of DLE-MGC technique under 2000 epochs.

**Figure 6:** Comparative accuracy analysis of DLE-MGC technique with recent methods.

**Table 1:** Music genre classification result analysis of DLE-MGC technique under 1000 epochs.

Epoch-1000				
Classes	Precision	Recall	F-score	Accuracy
Pop/Rock	94.87	93.86	94.70	95.87
Country	94.55	97.87	95.05	97.81
Electronic	93.17	95.60	96.27	93.56
R&B	94.18	97.34	96.37	94.94
Latin	97.76	99.16	97.75	97.03
Jazz	93.55	95.42	96.47	94.85
New age	94.31	95.75	94.40	93.72
Rap	96.45	97.12	96.01	97.06
International	92.27	93.42	96.76	93.59
Reggae	93.27	96.45	98.53	96.91
Folk	96.51	94.49	97.70	95.83
Vocal	98.78	95.65	98.47	95.06
Blues	94.94	95.46	96.41	94.27
Average	94.97	95.97	96.53	95.42

**Table 2:** Music genre classification result analysis of the DLE-MGC technique under 2000 epochs.

Epoch-2000				
Classes	Precision	Recall	F-score	Accuracy
Pop/Rock	95.98	95.58	97.00	95.98
Country	96.76	96.60	95.35	96.64
Electronic	94.42	96.51	97.32	96.14
R&B	95.68	95.44	97.63	95.59
Latin	94.69	95.40	95.78	94.78
Jazz	96.23	96.44	97.86	96.23
New age	96.55	96.26	97.38	96.31
Rap	96.93	95.51	97.43	95.72
International	96.45	95.86	95.32	96.08
Reggae	96.64	95.22	96.36	95.87
Folk	95.03	96.34	96.07	95.90
Vocal	96.34	96.68	97.82	96.45
Blues	94.27	95.29	95.91	94.64
Average	95.84	95.93	96.71	95.87

**Table 3:** Average classification result analysis of DLE-MGC technique.

Measures	Epoch-1000	Epoch-2000
Precision	94.97	95.84
Recall	95.97	95.93
F-score	96.53	96.71
Accuracy	95.42	95.87

**Table 4:** Accuracy analysis of DLE-MGC with existing techniques.

Methods	Accuracy
DLE-MGC	95.87
DBTMPE	94.27
Two-LSTM	64.88
P2-PQA	64.10

## Data Availability

The data used to support the findings of this study are available from the corresponding author on request.
